The article "Diagnosis of Prostate Cancer Using GLCM Enabled KNN Technique by Analyzing MRI Images" was retracted in 2024. Reasons: signs of a paper mill; suspected computer-generated content; unreliable results or conclusions; concerns about the data.

# Diagnosis of Prostate Cancer Using GLCM Enabled KNN Technique by Analyzing MRI Images

**DOI:** 10.1155/2023/3913351

**Published:** 2023-01-24

**Authors:** L. Anand, Shivlal Mewada, WameedDeyah Shamsi, Mahyudin Ritonga, Noza Aflisia, Prakash KumarSarangi, Moses NdoleArthur

**Affiliations:** ^1^Department of Networking and Communications, SRM Institute of Science and Technology, Chennai, India; ^2^Dept. of Computer Science, Govt. College, Makdone (Vikram University), Ujjain, India; ^3^Information Technology, Al-Mustaqbal University College, Babylon 51001, Iraq; ^4^Universitas Muhammadiyah Sumatera Barat, Indonesia; ^5^Institut Agama Islam Negeri Curup, Indonesia; ^6^Department of CSE (AI&ML) Vardhaman College of Engineering, Hyderabad, India; ^7^Department of Biomedical Engineering, School of Engineering Sciences, College of Basic and Applied Sciences, University of Ghana, Legon P. O. Box LG 54, Accra, Ghana

## Abstract

Cancer has a disproportionately large influence on the death rate of adults. A patient needs to get a diagnosis of their condition as quickly as is humanly feasible in order to have the greatest chance of surviving their sickness. Skilled medical professionals use medical imaging and other traditional diagnostic methods to search for clues that may indicate the presence of malignant tendencies inside the body. Nevertheless, manual diagnosis may be time-consuming and subjective owing to the wide range of interobserver variability induced by the enormous number of medical imaging data. This variability is caused by the fact that medical imaging data are collected. Because of this, the process of accurately diagnosing a patient could become more difficult. To execute jobs that included machine learning and the interpretation of complicated imagery, cutting-edge computer technology was necessary. Since the 1980s, researchers have been working on developing a computer-aided diagnostic system that would help medical professionals in the early diagnosis of various malignancies. According to the most recent projections, prostate cancer will be discovered in the body of one out of every seven men at some time throughout the course of their life. It is unacceptable how many men are being told that they have prostate cancer, and the condition is responsible for the deaths of a rising number of men every year. Because of the high quality and multidimensionality of the MRI pictures, you will also need a powerful diagnosis system in addition to the CAD tools. Since it has been shown that CAD technology is beneficial, researchers are looking at methods to improve the accuracy, precision, and speed of the systems that use it. The effectiveness of CAD technology has been shown. This research proposes a strategy that is both effective and efficient for the processing of images and the extraction of features as well as for machine learning. This work makes use of MRI scans and machine learning in an effort to detect prostate cancer at an early stage. Histogram equalization is used while doing the preliminary processing on photographs. The image's overall quality is elevated as a result. The fuzzy C means approach is used in order to segment the images. Using a Gray Level Cooccurrence Matrix (GLCM), it is feasible to extract features from a dataset. The KNN, random forest, and AdaBoost classification algorithms are used in the classification process.

The article "Diagnosis of Prostate Cancer Using GLCM Enabled KNN Technique by Analyzing MRI Images" was retracted in 2024. Reasons: signs of a paper mill; suspected computer-generated content; unreliable results or conclusions; concerns about the data.

## 1. Introduction

The prostate is a somewhat unremarkable organ in the human reproductive system, yet it plays an essential role. Sperms are carried throughout the male reproductive system by the fluid that is generated by the prostate gland and known as semen. It is situated between the urinary bladder and the upper urethra, which is the conduit via which urine is passed from the urinary bladder. Prostate cancer (PC) is the most common nonmelanoma cancer in men, and it has emerged as one of the most pressing issues facing public health on a worldwide scale. An uncontrolled growth of cells inside the prostate gland is what leads to the development of prostate cancer [1].

Cancers that originate in the peritoneal cavity may advance in one of two different ways, gradually or rapidly. The prostate is almost often the only organ that is affected by tumours with a sluggish growth rate. It is estimated that around 85 percent of all cases of pancreatic cancer are brought on by types of tumours that develop slowly. In the treatment of these circumstances, active monitoring is an absolutely necessary component [2]. The second kind of pancreatic cancer, in contrast to the first, grows swiftly and metastasizes to other areas of the body via a process called spread. Monitoring techniques that can be relied on are required in order to accomplish the task of differentiating between these two types of evolution. In most cases, the early detection of PCs is accomplished by the performance of routine physical tests. The first thing that has to be done in order to devise a treatment plan is to pinpoint the precise location of the prostate. In order to achieve a high survival rate, screening approaches that are both effective and dependable are used. The PSA test, transrectal ultrasonography, and magnetic resonance imaging (MRI) are the three types of prostate cancer screening that are being used the most often [3].

The primary focus of the initial set of recommendations was entirely on the categorization of clinical relevance; however, the primary focus of the modifications to the original prostate MR guidelines was on the development of worldwide standards for MRI. This is in direct opposition to the major focus that the first guideline placed on. The level of picture capture and reporting is meant to be kept up to date with each new release, which is the goal of this endeavour. Recent research has undertaken a number of studies that assessed the effect of proposals that were made based on these criteria. These investigations were done to explore recent research. For the purpose of classifying a clinically relevant PC lesion, any one of the following approaches may be utilized. When identifying lesions that are fairly small but rather severe, there are, nonetheless, some limits that must be taken into consideration. It has been shown that a PI-RADS guideline may be of assistance in the process of detecting cancer that has spread outside of the prostate, which is a factor that has a substantial impact on the staging of cancer. This is due to the fact that the sickness has spread to other parts of the body [4].

The article "Diagnosis of Prostate Cancer Using GLCM Enabled KNN Technique by Analyzing MRI Images" was retracted in 2024. Reasons: signs of a paper mill; suspected computer-generated content; unreliable results or conclusions; concerns about the data.

The biological databases include a tremendous amount of information for researchers to peruse [5]. It is getting more challenging to gain insights from the massive amounts of data that are being collected. Machine learning is a kind of learning in which a machine utilizes examples, comparisons, and past experience to improve itself. This type of learning came about as a result of the fact that data mining has become such an important component of knowledge mining. The fundamental concept behind machine learning is pattern recognition in data and the ability to draw quick conclusions based on a variety of different datasets. Using methods derived from machine learning, automated screening of ligand libraries may be carried out [6, 7].

Histopathology, which is used for the diagnosis and study of illnesses that damage the body's tissues, requires the careful examination of tissues and/or cells using a microscope. Histopathologists provide diagnoses based on the analysis of tissue samples in order to assist other medical professionals in the treatment of patients.

Through the examination of MRI images, the machine learning approaches that are presented in this article may identify prostate cancer. Histogram equalization is used during the preprocessing stage of image creation. It results in a higher overall picture quality. The fuzzy C means algorithm is used to carry out the process of image segmentation. The method known as the Gray Level Cooccurrence Matrix is used in order to extract features. The KNN, random forest, and AdaBoost classification algorithms are used in the process of classification.

The article "Diagnosis of Prostate Cancer Using GLCM Enabled KNN Technique by Analyzing MRI Images" was retracted in 2024. Reasons: signs of a paper mill; suspected computer-generated content; unreliable results or conclusions; concerns about the data.

## 2. Literature Survey

In order to accomplish the findings that they did, Rampun et al. [8] used a combination of an anisotropic diffusion filter and a median filter. Due to the fact that noise and edges both produce uniform gradients, it is more challenging to remove noise from photographs that have a low signal-to-noise ratio. A noise gradient can be recognized by using a thresholding technique, but the edges of the gradient are smoothed down. Samarasinghe et al. [9] stated that the researchers carried out their work with the use of a three-dimensional sliding Gaussian filter. Because this filtering strategy is unable to eliminate the noise distribution in MPMRI photos, more complex and innovative alternative strategies have been offered as a means of addressing these kinds of problems. MPMRI images make advantage of the sparsity that is provided by the wavelet decomposition, which means that these pictures may gain benefit from the wavelet decomposition and shrinking techniques. One example of an orthogonal transformation that may be seen in action is the wavelet transform. The Rician distribution, on the other hand, maintains the unwanted noise signal even when applied to the wavelet transform domain. As a consequence of this, the wavelet and scaling coefficients have to be adjusted in part due to the distribution of noise in the data. Therefore, in order to filter out the noise in T2W photos, Lopes et al. [10] used the joint detection and estimation approach. In order to calculate the noise-free wavelet coefficient, a maximum a posteriori estimate of the noisy wavelet coefficients is used. After being normalized, each picture was adjusted such that the PZ region had a mean value of one and a standard deviation of zero. After that, the normalized MPMRI pictures were used for the purposes of instruction and evaluation within the study. As a consequence of carrying out this method, the dynamic ranges of the various MPMRI sequence intensities have been brought into alignment, which has led to an increase in the segmentation stability.

Raw images are distorted not only by noise but also by a bias field that is produced by an endorectal coil [11]. Variation in signal intensity may be attributed to the bias field, which can be detected in MRI images. As a consequence of this, the intensity of similar tissues changes greatly depending on where they are located in the image. This causes succeeding stages of the computer-aided design system to be more challenging.

Because there is a learning component involved in both the process of segmentation and the process of classification, training images are necessary. Therefore, in order to make a diagnosis that is correct and can be performed automatically, it is essential to collect signal intensity images from patients whose readings are comparable to those of one another and who are members of the same group (cancerous or noncancerous). There is still some degree of variation in the photographs that are generated, even when all of the patients are examined with the same scanner, using the same technique, and using the same settings. Viswanath et al. [12] used the piecewise linear normalization strategy to normalize T2W photos in order to eliminate the variability across patients and assure repeatability. This was done in order to normalize the images. During the course of this inquiry, piecewise linear normalizing techniques were used in order to locate and extract the original foreground.

The article "Diagnosis of Prostate Cancer Using GLCM Enabled KNN Technique by Analyzing MRI Images" was retracted in 2024. Reasons: signs of a paper mill; suspected computer-generated content; unreliable results or conclusions; concerns about the data.

Atlas-based segmentation is the method that is employed the most often in medical image analysis. This is due to the fact that it works better with pixel intensities and regions that are poorly defined. When analyzing prostate data obtained from MRI, Tian et al. [13] used the graph cut segmentation strategy with the superpixel notion to get their desired results. Cut-and-paste segmentation is helpful since it reduces the amount of computing and memory resources that are required. Due to the fact that it is only partially automated, the procedure has to be set up manually. Martin et al. [14] separated the prostate from the MRI using an atlas-based deformable model segmentation technique. In order to move the contour closer to the borders of the prostate, an atlas-based technique was used, and a deformable model was used, a probabilistic depiction of the location of the prostate.

A totally automated technique for segmenting the prostate in MRI images was developed by Vincent et al. in paper [15]. This method made use of an active appearance model. Through the use of a multistart optimization process, the model is meticulously matched to the test photographs.

An atlas-based matching strategy was utilized by Klein et al. [16] to automatically segment the prostate. They did this by using a nonrigid registration and comparing the target image to a large number of prelabeled atlas photographs with hand segmentation. Following the completion of registration, the matching segmentation photographs are concatenated in order to provide an MR image segmentation of the prostate.

In order to accomplish segmentation of the prostate, deformable models make use of both internal and external energies. Internal energy is used to smooth the boundaries of the prostate, while external energy is used to propagate the shape. Chandra et al. [17] developed a method that can swiftly and automatically segment prostate images that were scanned without the use of an endorectal coil. During the training phase of this case-specific deformable system's initialization process, a patient-specific triangulated surface and image feature system is developed. The initialization surface of the picture may be changed with the help of an image feature system by using the concept of template matching. In recent years, there has been an increase in the use of multiatlas techniques and deformable models to the process of automatic prostate segmentation.

The article "Diagnosis of Prostate Cancer Using GLCM Enabled KNN Technique by Analyzing MRI Images" was retracted in 2024. Reasons: signs of a paper mill; suspected computer-generated content; unreliable results or conclusions; concerns about the data.

In the research carried out by Yin et al. [18], a prostate segmentation method that is both fully automated and very reliable was used. When a normalized gradient field has been cross-correlated with the prostate, the graph-search approach is used to enhance the prostate mean shape system. This helps to better understand how the prostate develops over time. Deformable models are helpful in situations when noise or sampling irregularities are to blame for the appearance of unwanted prostate boundaries.

The simplest strategy to achieve a comprehensive response while also overcoming challenges with segmentation is to make use of a technique that involves graph cutting. For the purpose of segmenting the prostate, Mahapatra and Buhmann presented the graph cut strategy [19], which makes use of the semantic information that was collected. Random forests were used as part of a super-voxel segmentation strategy in order to provide an estimate of the volume of the prostate as well as its location. The volume of the prostate was further optimized with the help of random forest classifiers that were trained on photos and the signals from its surroundings. In order to optimize the graph cuts used for prostate segmentation, a Markov random field is used.

Puech et al. [20] created a set of rules for predicting test results by making use of the data that was obtained via medical support systems. It is feasible to categorize data by making use of similarity measures and the fundamental method of supervised machine learning known as k-nearest neighbor (k-NN). The k-means clustering technique is an unsupervised algorithm that splits the data into k-numbers of groups in an iterative manner. k is the number of iterations. Every point in the feature space is given an identifier that corresponds to the k-number of centroids that is geographically closest to it. After that step has been completed, a new mean is calculated for each cluster, and the positions of each cluster's centroid are modified so that they are consistent with the new mean. The procedure of assigning and updating centroids will continue until such time as the centroids will no longer undergo any changes. The number of classes that make up a cluster is often denoted by the letter k.

The article "Diagnosis of Prostate Cancer Using GLCM Enabled KNN Technique by Analyzing MRI Images" was retracted in 2024. Reasons: signs of a paper mill; suspected computer-generated content; unreliable results or conclusions; concerns about the data.

The method of classification known as linear discriminant analysis (LDA) is used in order to establish an ideal linear separation between the two classes. This results in an increase in the difference between the interclasses and a decrease in the difference between the intraclasses. The Naive Bayes classifier is the one that is used most often. It is a probabilistic kind of classification since it is based on the assumption that each dimension of the features being analyzed is independent. Using this method, it is thus feasible to classify photographs with the greatest possible posterior probability.

Another widely used approach to classification is known as adaptive boosting, or AdaBoost for short. AdaBoost is an ensemble learning technique that was created in [21]. Using this approach, many weak learners are merged to produce a single powerful classifier. The AdaBoost (AdB) classifier is superior to the random forest classifier in terms of performance. This classifier gives preference to weak learners such as decision stumps, classification trees, and regression trees. During the course of their research, Lopes et al. used an AdaBoost classifier to complete the classification procedure.

Using Gaussian processes to label classes is one way to do class labelling within the context of an approach to classification that is based on a sparse kernel. This approach is known as the kernel strategy, and it derives its name from the fact that it generates new labels by making use of the whole training dataset. In order to assign a category to an unlabeled image, sparse kernel classification algorithms rely on a restricted number of samples that have been tagged from the dataset that is used for training [22]. The support vector machine (SVM), which is an example of a sparse kernel technique, is used to select the best linear hyperplane to split up into two label classes with the largest margin of error. This is accomplished by comparing the data to determine which linear hyperplane produces the best results. Choosing the most appropriate linear hyperplane on which to categorize the data enables this goal to be realised. Support vector machines are useful classifiers in applications that take place in the real world because they are trustworthy and can be extended. This makes them helpful in applications that take place in the actual world.

## 3. Methodology

This section presents machine-learning techniques for prostate cancer detection by analyzing MRI images. Image preprocessing is done using histogram equalization. It improves image quality. Image segmentation is performed using the fuzzy C means algorithm. Features are extracted using the Gray Level Cooccurrence Matrix algorithm. Classification is performed using the KNN, random forest, and AdaBoost algorithms.  Figure 1 shows the machine-learning techniques for prostate cancer detection by analyzing MRI images.

The article "Diagnosis of Prostate Cancer Using GLCM Enabled KNN Technique by Analyzing MRI Images" was retracted in 2024. Reasons: signs of a paper mill; suspected computer-generated content; unreliable results or conclusions; concerns about the data.

Pictures that are clearer and more detailed may be obtained from medical imaging procedures such as digital X-rays, MRIs, CT scans, and PET scans by using the basic image processing method of histogram equalization. For the purpose of determining the pathology and arriving at a diagnosis based on these pictures, high-definition photographs are required. After all of the processing is done, applying histogram equalization to the image will make any noises that were previously hidden in the picture audible again. This method is often used in the field of medical imaging analysis [23]. After determining the image's gray mapping by the use of gray operations, the approach generates a gray-level histogram that has levels of gray that are perfect, consistent, and smooth.

Clustering is a strategy that groups together patterns that are similar to one another in an effort to find the underlying links that exist between the pixels in a picture. This approach's goal is to uncover the underlying linkages that exist. The word “clustering” refers to the practise of grouping objects into groups based on the fundamental features they share with one another. When using the FCM approach, the data objects are sorted and categorized into groups based on the membership values that they have. During the process of maximising the function of the object, the technique of least squares is used, and the division of the final data is carried out once the computation has been completed [24].

Feature extraction is a method of image processing that may be used to lessen the amount of data stored on a computer by deleting dimensions from a collection of feature subsets that are deemed unnecessary or irrelevant. The GLCM approach is used to recover the properties of the texture and preserve a connection among the pixels. This is accomplished by calculating the cooccurrence values of the gray levels. The general linear model (GLM) is constructed by applying the conditional probability density functions p(i, j|d, ș) and the selected direction of ș = 0, 45, 90, or 135 degrees, and the distances *d* ranging from 1 to 5. The GLCM algorithm is used in order to accomplish this goal. For instance, the probability that two pixels with the same gray level I and/or j) are spatially connected may be found by using the function p(i,j|d,ș), and the distance in question is referred to as the intersample distance (*d*). The GLCM places a strong emphasis on contrast, correlation, energy, entropy, and homogeneity among its many significant qualities [25].

The article "Diagnosis of Prostate Cancer Using GLCM Enabled KNN Technique by Analyzing MRI Images" was retracted in 2024. Reasons: signs of a paper mill; suspected computer-generated content; unreliable results or conclusions; concerns about the data.

KNN is a kind of supervised method that is used particularly for classification purposes. When using this method, the most important thing to remember is that it always produces the same results, even when using the same training data. It is possible to give a class to all of the samples or only one or two of them based on the value that is closest to it in the population. The Euclidean distance is specified in the equation that was just presented as a way to quantify how similar two-pixel places are to one another. Therefore, the pixels wind up in the same group, which is where they should have been all along given the odds. In KNN, the letter K represents the neighborhood with the shortest distance between any two neighbors. The number of homes that are located close is the most essential consideration. If there are just two courses, the number of courses will almost always be an odd number. At that stage in the algorithm, the calculation known as the nearest neighbor calculation is *K* = 1. This is the simplest of all the conceivable scenarios to take place [26].

The model creates random forests, thus the name “random forest,” and this is precisely what it does. RF stands for “random forest.” With the help of this approach, it is possible to construct a forest of decision trees, each of which is educated in a distinct way. This method was used in the construction of the current forest of trees, which depicts all of the feasible responses to the questions including multiple choice options. As a direct consequence of this, they were included into the calculations in order to create even more accurate estimations [27].

There is a method known as AdaBoost that may be used to classifiers that are not very effective in order to increase the accuracy with which they classify data. The algorithm AdaBoost will be used to distribute the initial weights for each observation. After a few iterations, observations that have been incorrectly categorized will be given greater weight, while observations that have been successfully classified will be given less weight. The efficacy of the classifier is significantly improved as a result of the weights on the observations being measures of the class to which the observation belongs. This helps to decrease instances of incorrect categorization. When using the strategy of “boosting,” many pupils who are struggling academically are successively fitted in an adjustable manner. In each subsequent model in the series, observations that were given insufficient weight in earlier models are given a greater amount of emphasis in that model [28].

The article "Diagnosis of Prostate Cancer Using GLCM Enabled KNN Technique by Analyzing MRI Images" was retracted in 2024. Reasons: signs of a paper mill; suspected computer-generated content; unreliable results or conclusions; concerns about the data.

## 4. Result Analysis

In this experimental set up, PROMISE dataset [29] is used. 80 MRI images are used in the study. 55 images are used in training of model and 25 images are used for testing of model. Image preprocessing is done using histogram equalization. It improves image quality. Image segmentation is performed using the fuzzy C means algorithm. The Gray Level Cooccurrence Matrix technique is used in the process of feature extraction. The KNN, random forest, and AdaBoost classification algorithms are used in the classification process. Accuracy, sensitivity, and specificity are the three characteristics upon which the performance of a variety of distinct algorithms is evaluated and compared during the course of this research. Performance is shown in Figures 2–4. From the figures, it is clear that the accuracy, sensitivity, and specificity of KNN algorithm is better than AdaBoost decision tree and random forest algorithm. GLCM feature selection results in increasing accuracy of KNN technique.

## 5. Conclusion

Cancer is the leading cause of mortality among those over the age of 65. If a diagnosis of the patient's condition can be made as quickly as possible, it will significantly improve the patient's chances of surviving the illness. Medical imaging, much like traditional diagnosis, is analyzed by skilled specialists who search for any indicators that the body may be expressing malignant tendencies. These professionals seek for any signals that the body may be displaying cancerous tendencies. On the other hand, manual diagnosis may be time-consuming and subjective owing to the wide range of interobserver variability that is caused by the huge quantity of medical imaging data. This variability is a result of the vast amount of data that is included in medical images. Because of this, providing an appropriate diagnosis to a patient might be challenging. In order to accomplish tasks that required the use of machine learning and the processing of intricate pictures, it was necessary to make use of the most cutting-edge computer technology. Since many decades ago, efforts have been made to create a computer-aided diagnostic system with the intention of supporting medical professionals in the early diagnosis of various types of cancer. It is expected that one man in every seven will be diagnosed with prostate cancer at some point throughout their lives. An unacceptably high percentage of men are being told they have prostate cancer, and each year, this illness claims the lives of an increasing number of people. Due to the high quality and the multidimensional nature of MRI pictures, it is necessary to make use of a suitable diagnosis system in conjunction with CAD tools. I am now engaged in the process of developing a project that is based on the goals that we have in common. Because it has been shown that the computer-aided design (CAD) technology that is already in use is beneficial, researchers are presently focusing their efforts on creating strategies to increase the accuracy, specificity, and speed of these systems. This research presents a model that is effective with regard to the processing of images, the extraction of features, and the acquisition of new skills using machine learning.

The article "Diagnosis of Prostate Cancer Using GLCM Enabled KNN Technique by Analyzing MRI Images" was retracted in 2024. Reasons: signs of a paper mill; suspected computer-generated content; unreliable results or conclusions; concerns about the data.

## Figures and Tables

**Figure 1:** Machine-learning techniques for prostate cancer detection by analyzing MRI images.

**Figure 2:** Accuracy comparison of classifiers for prostate cancer prediction.

**Figure 3:** Sensitivity comparison of classifiers for prostate cancer prediction.

**Figure 4:** Specificity comparison of classifiers for prostate cancer prediction.

## Data Availability

The data shall be made available on request.
